# Planar Supported Membranes with Mobile SNARE Proteins and Quantitative Fluorescence Microscopy Assays to Study Synaptic Vesicle Fusion

**DOI:** 10.3389/fnmol.2017.00072

**Published:** 2017-03-16

**Authors:** Volker Kiessling, Binyong Liang, Alex J. B. Kreutzberger, Lukas K. Tamm

**Affiliations:** ^1^Center for Membrane and Cell Physiology, University of VirginiaCharlottesville, VA, USA; ^2^Department of Molecular Physiology and Biological Physics, University of VirginiaCharlottesville, VA, USA

**Keywords:** SNARE, supported membrane, fluorescence microscopy, TIRF, synaptic vesicle fusion

## Abstract

Synaptic vesicle membrane fusion, the process by which neurotransmitter gets released at the presynaptic membrane is mediated by a complex interplay between proteins and lipids. The realization that the lipid bilayer is not just a passive environment where other molecular players like SNARE proteins act, but is itself actively involved in the process, makes the development of biochemical and biophysical assays particularly challenging. We summarize *in vitro* assays that use planar supported membranes and fluorescence microscopy to address some of the open questions regarding the molecular mechanisms of SNARE-mediated membrane fusion. Most of the assays discussed in this mini-review were developed in our lab over the last 15 years. We emphasize the sample requirements that we found are important for the successful application of these methods.

## Introduction

Neurotransmitter release at the synapse, accomplished by the fusion of synaptic vesicles with the presynaptic membrane, is a fast and highly regulated Ca^2+^ dependent process that is catalyzed by the neuronal SNAREs synaptobrevin-2 (Syb2, VAMP-2), SNAP-25 and syntaxin-1a (Syx1a; Jahn and Scheller, 2006; Jahn and Fasshauer, 2012; Rothman, 2014). Despite tremendous progress in this field, we are still missing a molecular timeline that proceeds from docking of synaptic vesicles to the plasma membrane, through priming of the fusion machinery, and eventually to fusion of the two membranes once an action potential reaches the synaptic terminal (Jahn and Fasshauer, 2012; Südhof, 2013). In addition to SNAREs at the core of the fusion machinery, several protein players that regulate the fusion process have been identified and characterized. Munc18, a 68 kDa soluble protein, is essential for fusion (Hata et al., 1993; Verhage et al., 2000) and has been proposed to arrange the SNAREs within a larger acceptor complex (Ma et al., 2013; Baker et al., 2015). Munc13, a 196 kDa protein, is associated with priming of synaptic vesicles (Ma et al., 2013), while complexin (Cpx), a 15 kDa helical protein, has been identified as inhibitor of spontaneous, i.e., Ca^2+^ independent, vesicle fusion (Yang et al., 2010) as well as a facilitator of fast synchronized fusion (Xue et al., 2007; Maximov et al., 2009). Synaptotagmin 1 (Syt1), a 47 kDa membrane protein consisting of two C2 membrane binding domains, has been identified as the Ca^2+^ sensor for fast synchronized release in hippocampal neurons (Perin et al., 1990, 1991; Maximov and Südhof, 2005). The exact role of these proteins and the nature of the events that constitute the intermediates of the fusion machinery during docking, priming and onset of fusion are highly debated. While the importance of the above proteins could be assessed by innovative *in vitro* and *in vivo* experiments, the role of lipids and their interactions with proteins has not been explored in comparable detail. Recombinant protein in combination with model membranes has been an important tool to investigate membrane fusion *in vitro*. Starting with the initial SNARE-mediated liposome fusion assay introduced by Weber et al. (1998) and Rothman (2014) that helped formulate the current version of the “SNARE hypothesis”, reconstitution experiments that try to measure the fusion reaction itself have received a lot of attention. However, to dissect the molecular details of the docking, priming and fusion steps, the underlying affinities and concentration dependencies between subsets of the relevant proteins and lipids as well as their complex interactions should be mapped and quantitatively controlled. One route that we have taken over the last years is to exploit fluorescence microscopy assays in combination with planar supported membranes (Tamm, 1984; Tamm and McConnell, 1985). The planar geometry of the sample allows the application of sophisticated fluorescence microscopy methods to probe the dynamics, structure and function of lipids and proteins within the lipid bilayer (Tamm and Kalb, 1993). Starting with the necessary sample requirements and preparations, we will describe fluorescence assays that we developed and applied to address some of the puzzling questions that remain around the synaptic vesicle fusion mechanism.

## Sample Preparation

While a thorough discussion of this subject goes beyond the scope of this review, we want to emphasize some characteristics of the sample preparation techniques that we found were most important for meaningful applications.

### Supported Membranes

There are two fundamentally different techniques for supported lipid bilayer formation: direct vesicle fusion and a combined Langmuir-Blodgett transfer/vesicle fusion (LB/VF) method (Tamm, 1984; Kalb et al., 1992). Perhaps due to its simplicity, most research groups have employed the direct vesicle fusion method. However, integral membrane proteins in this type of bilayers are usually not laterally mobile, and membrane fusion observed in this system often does not reproduce physiological or other *in vitro* assays (Bowen et al., 2004; Fix et al., 2004; Liu et al., 2005). In the LB/VF method, first, a lipid monolayer is transferred from the air-water interface of a Langmuir trough onto a clean substrate, then liposomes that might contain protein fuse with this supported monolayer to form the second leaflet of the final bilayer (Figure 1A). Two properties of the resulting supported membrane are essential for the assays discussed below. First, reconstituted SNARE proteins are highly oriented with their cytosolic domain facing away from the substrate (Figure 1B). Consequently, they are highly mobile in the plane of the bilayer, even at relatively high protein to lipid ratios (Wagner and Tamm, 2001; Kiessling and Tamm, 2003; Liang et al., 2013). Second, the two step preparation procedures allow the assembly of asymmetric lipid bilayers (Crane et al., 2005; Kiessling et al., 2006). The LB/VF method can also be used to introduce a polymer cushion between substrate and supported membrane to increase mobility of large membrane proteins (Wagner and Tamm, 2000). It is important to point out that for SNAREs with their small C-terminal domain, this polymer is not required (Wagner and Tamm, 2001; Domanska et al., 2009). For a detailed discussion of the supported membrane preparation and its advantages see also two recent reviews (Kiessling et al., 2015a,b).

**Figure 1:** **Sample preparation and requirements for supported membrane—SNARE applications. (A)** Reconstitution of trans-membrane proteins into supported membranes is accomplished by a two-step technique. In step i, a lipid monolayer is transferred from the water-air interface of a Langmuir-Blodgett trough onto an appropriate hydrophilic substrate. In step ii, protein-containing liposomes are fused with the monolayer in a flow-through chamber to assemble the second leaflet of the supported bilayer and to incorporate membrane proteins. **(B)** Syntaxin-1a (Syx1a), reconstituted by the technique pictured in **(A)** is oriented with its SNARE motif facing away from the substrate. Incubation of labeled Syx1a (Alexa 546 at residue 192) with Co^2+^ results in ~90% fluorescence quenching while the same application with a symmetrically distributed rhodamine labeled lipid results in ~50% fluorescence quenching (Liang et al., 2013). **(C,D)** Formation of 1:1 Syx1a:SNAP-25 complex in DPC as demonstrated by ion-exchange chromatography and SDS-PAGE. Equal molar amounts of Syx1a and SNAP25 are mixed and incubated overnight in DPC before ion-exchange purification. **(C)** MonoQ elution profile: the blue trace shows UV absorption (left axis) and the red trace shows the eluted buffer conductivity (right axis). The red vertical lines at the bottom denote collected fractions, and fractions run on SDS-PAGE gels are labeled with corresponding capital letters. **(D)** SDS-PAGE of protein samples purified by MonoQ column chromatography. Since SNAP-25 is about twice the molecular mass of syntaxin (residues 183–288), the SNAP-25 band is twice as strong as the Syx1a band when they are in a molar ratio of 1:1 (Kreutzberger et al., 2016). **(A)** is reprinted from Kiessling et al. (2015a) with permission from Elsevier. **(C,D)** are reprinted from Kreutzberger et al. (2016) with permission from Elsevier.

### Membrane Proteins

Both Syb2 and Syx1a are integral membrane proteins which are anchored to vesicle or target membranes, respectively, through a single C-terminal transmembrane helix. Both proteins are prone to aggregation in membranes, especially Syx1a. The effect of Syx1a clustering in the membrane has been explored extensively and its biological implication has been a hotly debated topic (van den Bogaart et al., 2013). Although Syx1a is routinely purified with different types of detergents, including octyl-beta-glucoside, cholate, or CHAPS, we have recently discovered that dodecylphosphocholine (DPC) can ensure the monomeric form of Syx1a (Liang et al., 2013). Furthermore, by employing DPC during the assembly of a Syx1a:SNAP-25 acceptor complex, we are able to prepare this complex in a strict 1:1 stoichiometry, which results in a highly active acceptor SNARE complex (Figures 1C,D; Kreutzberger et al., 2016).

Nascent SNAP-25 is a soluble protein that becomes post-translationally modified and a peripheral membrane protein by palmitoylation of four cysteines in the linker region between the two SNARE motifs. Previously, most *in vitro* SNARE fusion studies have employed the soluble form of SNAP-25. We have engineered a quadruply dodecylated SNAP-25 through disulfide binding of a dodecyl methanethiosulfonate precursor to the four native cysteines of SNAP-25. This membrane-associated form of SNAP-25 can be employed to form a highly active target acceptor SNARE complex in liposomal or supported membranes that mediates fast and efficient fusion with Syb2-containing proteoliposomes (Kreutzberger et al., 2016).

For some of the fluorescence assays described here, labeling of membrane proteins with a fluorophore is an important aspect of sample preparation. Although membrane fusion can be observed with lipid and/or content labels, the labeling of the proteins themselves offer unique information, such as protein-protein interaction by FRET or membrane protein orientation by fluorescence interference contrast (FLIC). Protein labeling can be achieved through the genetic addition of a fusion protein, such as GFP, to the N- or C-terminus. Lately, thiol-reactive fluorophores have gained major attraction due to their small sizes, high quantum yield, photo stability, many color options and site-specificity by the relatively easy introduction of single cysteine mutations. The labeling efficiency of this reaction usually approaches unity if samples are handled in an oxygen-free environment. We have routinely labeled membrane proteins before the removal of their purification tags. The labeled samples are then rebound to the affinity medium and subjected to extensive washing to remove unreacted free labels (Liang et al., 2013).

## Measuring Interactions within Membranes by Fluorescence Recovery After Photo-Bleaching (FRAP) and Single Particle Tracking (SPT)

How does the lipid content of membranes interact with their protein content? This is probably the central question for determining what leads to membrane fusion during exocytosis. Systematic measurements of the diffusion behavior of lipids and proteins in membranes is one technique that can elucidate some of these critical interactions.

### Diffusion of Integral Membrane Proteins

Observing the recovery of fluorescent content in a certain membrane region which was depleted of all or most fluorescence by application of a strong laser pulse is a standard method to probe transport or diffusion mechanisms in biological and model membranes. The planar geometry of supported membranes make them especially suitable for patterned fluorescence recovery after photo-bleaching (FRAP; Figure 2A), an easy to apply and analyze version of FRAP that allows the determination of mobile fractions and diffusion coefficients (Smith and McConnell, 1978; Tamm and Kalb, 1993).

**Figure 2:** **Supported membrane—fluorescence microscopy assays. (A)** Fluorescence recovery after photobleaching (FRAP) records the recovery of fluorescence due to lateral diffusion in a region of interest in the membrane after application of a strong laser pulse. The total intensity of an area is recorded before and after the bleach pulse has been applied (Smith and McConnell, 1978). The example graph on the right shows the recovery of Alexa488 labeled t-SNAREs in supported membranes (Wagner and Tamm, 2001). **(B)** Single particle tracking (SPT). The movement of membrane components labeled with a single fluorophore are tracked within the *x*/*y* plane of the lipid bilayer. The statistically analysis of the trajectories can quantify the lateral mobility as well as reveal different modes of diffusion (Schmidt et al., 1995; Kiessling et al., 2006; Vasquez et al., 2014). The example image on the right shows single Alexa647 labeled t-SNAREs in inverse contrast. Movies of the moving protein can be seen on the original publisher’s website (Domanska et al., 2009). **(C)** Binding assay using total internal reflection (TIRF) microscopy. A totally reflected laser beam produces an exponentially decaying electric field at the glass/water interface. Fluorescent molecules or organelles that bind at the membrane surface increase the observable fluorescent intensity I over time (Kalb et al., 1989). Binding isotherms can be determined with various ligand concentrations and acceptor densities. Data on the right shows SNARE-specific binding of Alexa546 labeled Syb2(1-96) to a supported membrane (Domanska et al., 2009). **(D)** Single vesicle fusion TIRF assay. Fluorescence originating from the membrane (red, I_M_) or the content (green, I_C_) of single vesicles can be imaged when they enter the evanescent field of a TIRF microscope (Fix et al., 2004; Domanska et al., 2009). Characteristic intensity traces from docking vesicles can be analyzed to determine docking and fusion efficiencies as well as fusion kinetics (Kiessling et al., 2015b). Data on the right shows fluorescence originating from the membrane and content during a single vesicle fusion event (Kiessling et al., 2015a). **(E)** Distance measurements by FLIC microscopy. A Si/SiO_2_ substrate with different steps is used to probe the interference pattern originating from reflected excitation and emission light (Braun and Fromherz, 1997). Fitting the optical theory to the measured intensities I from different SiO_2_ layers allows the determination of the distance of specifically labeled protein residues from the lipid bilayer surface (Lambacher and Fromherz, 2002; Kiessling and Tamm, 2003). Data on the right shows a FLIC curve obtained from Alexa546 labeled Syx obtained under the same conditions as published in Liang et al. (2013). Data in **(A)** is reprinted from Wagner and Tamm (2001) with permission from Elsevier. Data in **(B,C)** was originally published in Domanska et al. (2009), © the American Society for Biochemistry and Molecular Biology. Data in **(D)** is reprinted from Kiessling et al. (2013) with permission from Elsevier.

In the first supported membrane assays with reconstituted SNARE proteins, Wagner and Tamm (2001) measured the diffusion of Alexa 488 labeled t-SNAREs at different concentrations of the anionic lipids phosphatidylserine (PS) and phosphatidylinositol-4,5-bisphosphate (PIP_2_). While the protein is highly mobile at relatively high concentration (l/p 400) in pure phosphocholine bilayers, increasing amounts of PS or PIP_2_ render large portions of t-SNAREs immobile. The lipid content, although to a lesser degree, also gets partially immobilized. Noteworthy is the much stronger effect that PIP_2_ has on lipid and protein mobility compared to PS indicating a strong interaction between PIP_2_ and the t-SNARE Syx1a. While the exact reason for the observed PIP_2_ and PS dependence of the mobility hasn’t been determined, it was later found that Syx1a clustering in model membranes also depends strongly on the lipid environment, especially on the cholesterol, PS and PIP_2_ content (Murray and Tamm, 2009; van den Bogaart et al., 2011).

### Diffusion of Peripheral Membrane Protein Domains

Progress in imaging technology over the last 20 years, especially in electron multiplying charged coupled devices (EMCCD) and the latest complementary metal oxide semiconductor (CMOS) cameras, allows the tracking of individually labeled molecules. Again, the planar geometry of the supported membrane simplifies the measurement and interpretation of molecule trajectories in or at the membrane (Figure 2B). We routinely use single particle tracking (SPT) to confirm the mobility of reconstituted membrane proteins (Domanska et al., 2009).

Synaptotagmins are the calcium sensors of exocytotic neurotransmitter release. Their two C2 domains interact with the lipid bilayer in a calcium dependent fashion which successively triggers membrane fusion and pore opening through a still debated mechanism. A detailed characterization of the C2 domain-lipid interactions is therefore of great interest. Vasquez et al. (2014) used SPT to study the diffusion behavior of single and tandem C2 domains of Syt7, the calcium sensor that triggers slow asynchronous release (Schonn et al., 2008). Their results are consistent with C2 domains that interact independently with the lipid bilayer, which is in contrast to Syt1, the calcium sensor for fast synchronous release, for which inter-domain cooperativity had been reported (Sun et al., 2007).

## Total Internal Reflection Fluorescence (TIRF) Microscopy

The planar geometry of supported membranes make them an excellent candidate for the application of total internal reflection fluorescence (TIRF) microscopy, where a beam of light gets totally reflected at the interface between the (glass-) substrate and water (Axelrod et al., 1983). Fluorescent molecules get excited by the evanescent electric field that decays exponentially, typically with a characteristic penetration depth of ~100–200 nm.

### Interactions with the Membrane: Binding

Supported membranes and TIRF microscopy are the ideal platform to record kinetic binding curves or binding isotherms of proteins and other membrane interacting molecules (Figure 2C; Kalb et al., 1990). The soluble cytosolic fragment of Syb2 tagged with green fluorescent protein (GFP) was shown to specifically bind to supported membranes containing reconstituted t-SNAREs. The resulting ternary SNARE complex could then be dissociated by the addition of NSF, α-SNAP and ATP mimicking the physiological SNARE assembly and disassembly cycle (Wagner and Tamm, 2001). These experiments represent the first functionally successful reconstitutions of SNARE proteins in supported membranes described in the literature. Binding studies with the soluble C2 domains of Syt and phase separated asymmetric supported bilayers revealed a preference of these domains in binding to liquid-disordered lipid domains that are enriched in anionic lipids over liquid-ordered domains. The same study also showed that Ca^2+^ dependent binding of C2 domains can change the lipid partitioning between the two phases (Wan et al., 2011). Reconstituting Syt1 into a planar bilayer allowed monitoring the Ca^2+^ and concentration dependent capture of negatively charged liposomes (Lu et al., 2014). Planar bilayers have also been used to investigate the role of the protein calcium activated protein for secretion (CAPS) on docking of Syb2 containing liposomes. CAPS, which has also been implied with docking and priming, promoted increased binding of Syb2 liposomes to planar bilayers containing PIP_2_ and Syx1a (James et al., 2009).

### Membrane-Membrane Interactions: Single Vesicle Fusion

The gold standard for *in vitro* SNARE experiments is to mimic the physiological vesicle fusion reaction itself. Single vesicle experiments have received increasing attention because they allow the independent observation of the initial docking event from the actual fusion event. While single vesicle assays can be implemented with immobilized proteoliposomes (Yoon et al., 2006; Kyoung et al., 2011; Diao et al., 2013), here, we will only discuss vesicle-supported membrane fusion assays (Figure 2D). The different types of commonly used single vesicle fusion assays have been discussed in Kiessling et al. (2015a).

Initial attempts of single vesicle to planar supported bilayers fusion assays resulted in fusion reactions that did not require SNAP-25 (Bowen et al., 2004; Liu et al., 2005), were Ca^2+^ dependent in the absence of Syt (Fix et al., 2004) or resulted in vesicle rupture instead of fusion (Wang et al., 2009). In all these experiments the direct vesicle fusion supported membrane preparation method was used and it raised the question if supported membranes were at all suited for SNARE-mediated fusion assays. Utilizing supported membranes prepared by the two-step LB/VF method, we could record fusion events that mimic the physiological SNARE requirement. Here, docking depends on the presence of Syx1a and SNAP-25 in the supported membrane and fusion occurred within tens of milliseconds (Domanska et al., 2009). The fusion reaction was followed by the transfer of fluorescently labeled lipids from Syb2 containing liposomes into the planar membrane. The fast change (~8 ms) of the fluorophores’ dipole orientation relative to the polarization of the evanescent field when the labeled lipids transfer from the spherical vesicle membrane to the planar supported membrane creates a signature signal for the onset of fusion (Kiessling et al., 2010) that can be used to accurately determine the fusion kinetics. Analysis of the fusion kinetics measured in a 1-palmitoyl-2-oleoyl-sn-glycero-3-phosphocholine (POPC)/cholesterol lipid environment revealed that eight parallel reactions had to take place between docking of vesicles and the onset of fusion (Domanska et al., 2009). It is plausible that these reactions are the formation of eight SNARE complexes at the fusion site. Karatekin et al. (2010) later found similar requirements for the number of SNAREs, although the experimental conditions were very different. In that work, a very low concentration of t-SNAREs were reconstituted into a polyethylene-glycol (PEG) containing supported membrane and the fusion delay times were simulated with a diffusion reaction model. We later showed that the fusion kinetics strongly depend on the lipid environment. Systematic introduction of up to 30 mol% phosphoethanolamine (PE) and 5 mol% PS into the vesicle and/or the supported membrane reduced the number of parallel reactions, i.e., the number of necessary SNARE complexes to 3 (Domanska et al., 2010). The variability of the SNARE cooperativity in purely SNARE mediated membrane fusion was further examined by combining bulk and single vesicle fusion assays. While small (~40 nm) highly curved liposomes were fusogenic with only one Syb2/liposome, large (~100 nm) liposomes needed 23–30 Syb2/liposome for efficient fusion (Hernandez et al., 2014). Observing the transfer of content dye from liposomes to the small cleft between substrate and supported membrane confirmed productive fusion (Kiessling et al., 2013) and allowed the easy distinction between full- and hemi-fusion events. Increasing amounts of cholesterol in either the supported membrane or the vesicle membrane shift the balance from unproductive hemi-fusion to productive full-fusion (Kreutzberger et al., 2015) and might increase the stability of the fusion pore (Stratton et al., 2016). While cholesterol can influence membrane fusion in many different ways (Yang et al., 2016), we attributed our observation to the stabilization of intermediates by the intrinsic curvature of cholesterol (Kreutzberger et al., 2015). The physiological relevance of this assay was validated when we employed a hybrid system consisting of purified synaptic vesicles from rat brain and a supported membrane containing recombinant plasma membrane SNAREs. Synaptic vesicles and liposomes containing Syb2 and Syt1 showed increased fusion efficiencies in the presence of Ca^2+^ and anionic lipids (Kiessling et al., 2013).

## Probing Protein Conformations in the Membrane: Fluorescence Interference Contrast (FLIC) Microscopy

FLIC microscopy is an interferometric fluorescence microscopy method that measures the distance of a planar fluorescent layer normal to a reflective interface and was originally developed to measure the distance of adhering cell membranes from a substrate (Lambacher and Fromherz, 1996; Braun and Fromherz, 1997, 1998). The interference contrast originates from the excitation and emission lights from fluorophores in front of a mirror at different distances. In practice, the mirror is implemented by the Si/SiO_2_ interface of a patterned Si wafer (Braun and Fromherz, 1997, 1998; Kiessling and Tamm, 2003; Liang et al., 2013). Once the sample is prepared on the FLIC substrate a relatively simple epifluorescence microscope with a lamp as excitation source is sufficient to record the images from which the intensities of the different terraces are extracted (Figure 2E). The optical theory that takes into account the spectra of excitation and emission of microscope, detector and fluorophore, the numerical aperture of the objective, the dipole orientation and quantum yield of the fluorophore, and the optical layer system that includes the supported membrane is fit to the data in order to get the desired z-distance (Lambacher and Fromherz, 2002). The accuracy of the resulting z-distance is determined by systematic errors caused by assumptions or measurements of the different optical layer thicknesses (oxide, water layer, membrane) and statistical errors caused by the fit and sample inhomogeneity.

Although the first application of FLIC was still limited by the available substrates and the relatively large size of the label, the distance of a N-terminus GFP label in a Syb2 construct within a SNARE complex was consistent with the crystal structure of a cis-SNARE complex published later (Kiessling and Tamm, 2003; Stein et al., 2009). More recently we utilized Alexa labeled proteins to perform site-directed FLIC microscopy. Different label positions allow the determination of an accurate picture of the orientation of the protein with respect to the lipid bilayer. With these bright labels the uncertainty of the absolute distance lies in the order of 1–2 nm. Distance changes that might occur after the protein of interest interacts with ligands that have been added to the sample, can be measured with sub 1 nm accuracy.

When reconstituting labeled integral plasma membrane proteins, we can take advantage of the supported membrane preparation procedure described above to achieve correctly oriented proteins as well as asymmetric lipid compositions between the two leaflets of the bilayer. Recently, by determining the distances of two residues at the N-terminus or the center of the Syx1a SNARE motif from the membrane surface, we showed that the cytoplasmic domain of monomeric Syx1a lies at the bilayer surface. Interestingly, complex formation within a stabilized acceptor SNARE complex consisting of Syx, SNAP25 and Syb2(49–96) or within a ternary SNARE complex results in a more upright position (Liang et al., 2013).

## Outlook

To solve the long-standing questions about how the secretory vesicle fusion machinery achieves its precise and reliable function, many different approaches must be utilized. A lot has been learned about the molecular requirements from *in vivo* and cell experiments and many mechanistic pictures have been drawn based on atomic resolution structures of soluble proteins or protein fragments. However, we need carefully controlled *in vitro* reconstitution experiments that are performed in the presence of defined lipid bilayers to gain further insights. The above discussed fluorescence assays with supported membranes are, in our view, among the most promising routes forward because they can deliver quantitative biochemical and functional data as well as structural information without neglecting important characteristics of the biological membrane like protein orientation, mobility and lipid asymmetry. Correlating the results of these different assays and considering that the samples with almost identical conditions can be prepared for a range of different structural and functional assays further enhances their value. We are very optimistic that the described approaches will soon deliver significant contributions to solve many of the remaining mysteries about the precise molecular interactions that underlie the mechanism of Ca^2+^-triggered exocytosis and synaptic vesicle fusion.

## Author Contributions

VK, BL, AJBK and LKT wrote the article.

## Funding

NIH grant P01 GM72694.

## Conflict of Interest Statement

The authors declare that the research was conducted in the absence of any commercial or financial relationships that could be construed as a potential conflict of interest.
